# Nanoparticles for Oral Cancer Diagnosis and Therapy

This article has been retracted.

**DOI:** 10.1155/2021/9977131

**Published:** 2021-04-23

**Authors:** Weiping Zheng, Qihui Zhou, Changqing Yuan

**Affiliations:** ^1^Department of Stomatology, The Affiliated Hospital of Qingdao University, Qingdao 266003, China; ^2^School of Stomatology, Qingdao University, Qingdao 266003, China; ^3^Institute for Translational Medicine, The Affiliated Hospital of Qingdao University, Qingdao University, Qingdao 266021, China

## Abstract

Oral cancer is the sixth most common malignant cancer, affecting the health of people with an unacceptably high mortality rate. Despite numerous clinical methods in the diagnosis and therapy of oral cancer (e.g., magnetic resonance imaging, computed tomography, surgery, and chemoradiotherapy), they still remain far from optimal. Therefore, an urgent need exists for effective and practical techniques of early diagnosis and effective therapy of oral cancer. Currently, various types of nanoparticles have aroused wide public concern, representing a promising tool for diagnostic probes and therapeutic devices. Their inherent physicochemical features, including ultrasmall size, high reactivity, and tunable surface modification, enable them to overcome some of the limitations and achieve the expected diagnostic and therapeutic effect. In this review, we introduce different types of nanoparticles that emerged for the diagnosis and therapy of oral cancers. Then, the challenges and future perspectives for nanoparticles applied in oral cancer diagnosis and therapy are presented. The objective of this review is to help researchers better understand the effect of nanoparticles on oral cancer diagnosis and therapy and may accelerate breakthroughs in this field.

## 1. Introduction

Oral cancer is the sixth most common malignant tumor around the world, and the 5-year survival rate is approximately 50% [1]. This disease tends to spread rapidly and is often capable of invading adjacent tissue and metastasis. Oral cancer could cause chronic pain, altered facial appearance, paraesthesia, dysfunction in speech, and dysphagia, as well as social isolation and psychological distress [2]. Oral cancer occurs because of genetic mutations that control cell cycles and is usually associated with excessive alcohol intake and tobacco use [3, 4]. Lengthy and expensive diagnostic strategies often lack the ability to efficiently differentiate between normal and tumor tissue, which could delay the initiation of treatment. In addition, the traditional treatment of oral cancer, such as surgery, radiotherapy, and chemotherapy, has certain limitations and side effects [5]. Thus, it is crucial to increase the effectiveness of diagnosis and reduce the side effects of treatment.

Recently, it has been demonstrated that biomaterials with unique (bio)physicochemical properties could mediate cell behaviors and even treat diseases, repair bodily functions, or regenerate tissues [6–15]. Particularly, the development of nanomaterials and their extensive application in diagnostic/therapeutic biomedicine has received much attention [16–23]. It is practicable to overcome conventional limitations of diagnosis and therapy with various nanoparticles (NPs) because of the particular anatomy and pathophysiological conditions of the tumor, such as angiogenesis, hypoxia, low extracellular pH, and lack of lymphatic drainage [24]. Tumor blood vessels are abnormal and highly porous, presenting spaces between endothelial cells [25, 26]. The macromolecules can specifically accumulate in the interstitial space of the tumor along with a large amount of blood plasma leakage and are not rapidly cleared, which is named enhanced permeability and retention (EPR) effect [27]. Nowadays, most NPs are being designed for the diagnosis and treatment of cancer based on the EPR effect by passive targeting. Considering the indetermination of EPR effect in the tumor microenvironment, more accurate and efficient active targeting strategies are needed. Therefore, NPS can be conjugated with ligands or antibodies to distinguish tumor-specific receptors, such as antiepidermal growth factor receptor (anti-EGFR) [28]. This enhanced targeting leads to decreased systemic toxicity and successful delivery. NPs can deliver not only the contrast agents which are helpful in imaging but also the active drug of chemoradiotherapy, as well as photosensitizers (PS) of photodynamic therapy (PDT) [29]. Besides, a variety of NPs exhibit unique controlled optical, magnetic, and electrical properties to generate light and heat for the diagnosis and therapy of oral cancer [30]. Moreover, an emerging nanotechnology-based methodology including biosensors [29, 31] and gene therapy [32] has given hope for cancer diagnosis and treatment. NPs including organic NPs (e.g., liposomes, dendrimers, and polymeric NPs) and inorganic NPs (e.g., gold NPs, magnetic NPs (MNPs), quantum dots (QDs), and carbon nanotubes) [33] have been widely used towing to their ultrasmall size, high reactivity, and tunable functional modification [34, 35]. This review summarized recent advances in the design of various NPs and their application in oral cancer diagnosis and treatment (Figure 1). Next, the challenges and future perspectives for NPs applied in oral cancer diagnosis and therapy are presented. This review is expected to help researchers better understand the effect of NPs on oral cancer diagnosis and therapy as well as may accelerate breakthroughs in this field.

## 2. Liposomes for Oral Cancer Diagnosis and Therapy

Liposomes are closed spherical particles made of amphiphilic phospholipid bilayers possessing a hydrophilic center. Hydrophilic or hydrophobic payloads can be encapsulated either within the hydrophilic center or within the lipid bilayer, respectively (Figure 2(a)). Liposomes were delivered into tumor tissue through passive targeting based on the EPR effect. Furthermore, to selectively target, ligands are attached to the liposome surface. For instance, high-affinity folate-bound liposomes can target folate receptors on the tumors selectively (Figure 2(b)) [36]. Different liposomal formulations had significant differences in stability characteristics and encapsulation efficiency, which can be employed to achieve unique diagnostic and therapeutic needs (Figure 2(c)) [37].

### 2.1. Liposomes for Oral Cancer Diagnosis

Liposomes have been widely used in the study of a cancer diagnosis. For instance, labeling with radionuclides such as ^64^Cu has commonly been achieved by the conjunction of the radionuclide and an anchor molecule present inside the hydrophilic center or encapsulated in the phospholipid bilayer. Mahakian et al. have proposed that ^64^Cu liposomes have the potential to detect early tumors compared to ^18^F-FDG [38].

### 2.2. Liposomes for Oral Cancer Therapy

Liposomes are used extensively in the delivery systems for a variety of anticancer agents to increase the efficacy of anticancer drugs and decrease the adverse effect. However, drug-loaded liposomes are easily cleared by the reticuloendothelial system (RES); therefore, many biocompatible polymers such as polyethylene glycol (PEG) have been employed for coating the surface of liposomes. The PEG is a synthetic hydrophilic polymer that can be crosslinked with the liposome surface to avoid RES clearance and increase the half-life in the blood circulation. Formulations prepared by loading antitumor drugs such as doxorubicin into liposomes are widely studied. El-Hamid et al. have proposed that PEGylated liposomal doxorubicin (PLD) has exerted a higher apoptotic effect on CAL-27 cells than free doxorubicin [39]. However, although PLD has good safety, long-term use in some patients has been related to the development of OSCC or precancer lesion [40, 41]. Other drugs incorporated in the liposomes include curcumin, paclitaxel, carboplatin, and cisplatin, which are also more effective to induce the apoptosis of cancer cells [42]. Two or more anticancer drugs with supplements were found to improve the efficacy of chemotherapeutic drugs. For example, the coencapsulated liposomal formulation of doxorubicin (Dox) and resveratrol (Res) has been studied in oral cancer, and drug combination has shown better efficacy in the treatment of oral cancer when tested *in vitro* [43]. Meanwhile, liposome-based formulations for gene therapy have great potential for oral cancer treatment. Liposomes constitute a promising alternative to viral vectors and provide a simple means of transferring therapeutic genes into target cells [44, 45]. Figueiredo et al. have formulated liposomes for the delivery of p12 to negatively regulate growth and inhibit tumor cell proliferation. *In vitro* cytotoxicity studies on the resistant mouse squamous cell carcinoma VII (SCC-VII) cells showed that this liposome formulation had greater cytotoxicity for cancer cells than naked DNA or other nonviral formulations [46].

Liposomes have also been explored as radionuclide carriers for tumor radiotherapy. Loading ^186^Re into the liposomes can effectively treat oral cancer with minimal side effects after convection-enhanced delivery [47]. Boron neutron capture therapy (BNCT), which is a tumor-targeting treatment modality based on the preferentially selective uptake of ^10^B target species by tumor cells and neutron irradiation, has attracted great interest for the effective elimination of tumor cells. Heber et al. have described a BNCT study mediated by a boron-rich liposomal system in the hamster cheek pouch oral cancer model. The liposomes could selectively deliver ^10^B agents to the tumor tissue, and then, neutron irradiation was given. The capture reaction between neutrons and ^10^B atoms gives rise to short-range particles and has a high relative biological effectiveness, resulting in substantial inhibition of tumor cell growth [48, 49].

PDT is a novel treatment that uses light to activate photosensitizers (PS) in the presence of oxygen, which then results in the generation of reactive oxygen species (ROS) [50]. Conjugation of the PS to the liposome can be used in PDT of cancer [51]. For example, Piskorz et al. have loaded liposomes with three porphyrazines containing annulated diazepine rings. Thereinto, magnesium(II) tribenzoporphyrazine has shown the highest photochemical properties and generated abundant singlet oxygen to reveal the highest phototoxic effect in oral squamous cell carcinoma lines [52]. Photochemical internalization (PCI) is a novel therapeutic method based on the fact that an anticancer drug and a PS may colocalize in the endolysosomal vesicles of cancer cells and anticancer drug release into the cytosol because of the light-induced damage to the membranes of vesicles. In this context, Peng et al. have found that liposomal formulation enhanced the toxicity of BLM on head and neck cancer cell lines when PDT was performed before BLM administration [53]. Furthermore, Gusti-Ngurah-Putu et al. have found that the administration of PDT before chemotherapy increased the nanoparticle uptake because of the increase of blood vessel permeability [54]. In addition, the embedding of PS in liposomes improves their phototoxicity, and the effect of phototoxicity is dependent on the cell type [55].

## 3. Dendrimers for Oral Cancer Diagnosis and Therapy

Dendrimers are three-dimensional, multibranched, and tree-like structures, which consist of three major components: a central core, repeated branches, and terminal functional groups (Figure 3(a)) [56]. Generally, the divergent method and the convergent method are mainly used to synthesize dendrimers. Up to now, dendrimers have been widely used in many areas, e.g., electrochemistry, drug delivery, and gene transfection.

### 3.1. Dendrimers for Oral Cancer Diagnosis

Dendrimers are attractive devices for the diagnosis of oral cancers. Wei et al. have developed DNA-dendrimer and polypyrrole (DDPpy) sensors to detect biomarkers of oral cancer, such as interleukin-8 RNA, interleukin-8 protein, and interleukin-1*β* protein, exhibiting higher specificity and better bioaffinity [58].

### 3.2. Dendrimers for Oral Cancer Therapy

Drugs are encapsulated in the interior cavity or are conjugated covalently to the terminal functional groups. Thus, dendrimers are widely used as promising drug delivery candidates. Ward et al. have coencapsulated methotrexate (an anticancer drug) and folic acid (FA, a targeting agent) in acetylated generation 5 dendrimer and reported tumor control better than free drug when performed on xenograft tumor growth models [59]. One step further may be the transfection of gene agents. Liu et al. have demonstrated polyamidoamine (PAMAM) dendrimer-mediated shRNAs can successfully silence human telomerase reverse transcriptase (hTERT) on oral squamous cell carcinoma (OSCC) cells and xenograft mouse models, suggesting the efficiency of this system in cell apoptosis and tumor growth inhibition [60]. Meanwhile, the use of FA-decorated PAMAM dendrimer generation 4 would result in improved gene transfection [61, 62]. Blockade of Src kinase activity by saracatinib-loaded dendritic nanoparticles (Nano-sar) effectively suppressed invasion and metastasis of head and neck squamous cell carcinoma (Figure 3(b)) [57].

## 4. Gold Nanoparticles for Oral Cancer Diagnosis and Therapy

Gold NPs have created widespread interest in biomedicine due to their good biocompatibility, ready bioconjugation, and high tissue permeability. Besides, they can be easily prepared and have precisely controllable size, high colloidal stability, and tunable optical properties [63]. Gold NPs in the nanometer size range have diverse geometries, such as nanospheres, nanorods, nanoshells, nanocages, and nanoprisms (Figure 4(a)) [64]. It is very critical to selectively transfer enough gold NPs to tumor tissue for accurate diagnosis or treatment. The EPR effect (so-called “passive targeting”) renders gold NPs accumulation in the tumor site, and then, they get into cells by the endocytosis process, which is mostly dependent upon their nanoscale. However, the uptake of gold NPs by passive targeting is relatively lower. Gold NPs conjugated to antibodies are worth considering for getting into the cell by active targeting [65]. El-Sayed et al. have demonstrated that anti-EGFR-antibody-conjugated gold NPs have a distinct difference in the distribution that conjugated NPs bind uniformly and specifically to the surface of the cancer cells *via* target cell recognition and bind nonspecifically and randomly to noncancerous cells [28].

### 4.1. Gold Nanoparticles for Oral Cancer Diagnosis

Cellular imaging by electron microscopy provides cellular labeling and anatomic details important for the early diagnosis of oral cancer. Gold NPs have highly controlled optical properties and can strongly scatter near-infrared (NIR) and visible light upon the irradiation of their surface plasmon resonance (SPR). This scattering of light that is much brighter compared with chemical fluorophores may be captured under dark-field microscopy and used to diagnose oral cancer [66]. Combining gold NPs and other materials can establish multifunctional nanoplatforms, which can be useful for cellular imaging. In the last few decades, gold NPs have received in-depth research in many diagnostic applications. Gold nanorods conjugated to anti-EGFR monoclonal antibodies can discriminate benign from premalignant and malignant oral lesions [67]. Gold NPs can be used in air scanning electron microscopy to highly improve tumor margins determination [68]. Matrix metalloproteinase 2 sensing upconversion NPs conjugated to gold NPs may serve as a diagnostic tool for monitoring the cancer cells *via* dynamic imaging [69]. Gold NPs can also be labeled as non-plasma-scattering probes for multiple dark-field imaging of live cancer cells [70]. Meanwhile, acid-transforming gold nanoclusters can be applied in optical coherence tomography (OCT) for detecting early-stage cancer [71]. The surface-enhanced Raman spectroscopy (SERS) technique is considered a convenient and noninvasive method for OSCC diagnosis [72]. Xue and Wang have proved that the SERS technique can be applied to analyze and discriminate the OSCC and even the different stages of the tumor. Gold NPs can enhance the intensities of the SERS spectrum enormously when they were added to the serum sample [73]. A customized gold-NP-reduced graphene-oxide- (AuNPs-rGO-) based bioelectrode has been prepared as an immunosensing platform for electrochemical detection of oral cancer [74]. Besides, gold NPs have contributed remarkably in improving the limit of detection (LOD) in conventional enzyme-linked immunosorbent assay (ELISA) protocol. For example, Chakraborty et al. have developed a gold-particle-based ELISA system for osteopontin (overexpressed in tongue tumors) detection, which exhibited high sensitivity [75].

### 4.2. Gold Nanoparticles for Oral Cancer Therapy

Gold NPs are widely applied as drug carriers in the therapy of oral cancer. Rathinaraj et al. have revealed folic acid-gold-bilirubin (FGB) NPs as a system to induce cell apoptosis through active targeting mediating folic acid and delivering bilirubin (a potential anticancer agent) to tumor sites, inducing ROS generation and DNA damage and altering the mitochondrial membrane potential [76]. Mackey and El-Sayed have shown that gold NPs can enhance 5-fluorouracil drug efficacy in HSC-3 cells *via* chemosensitization [77]. Gold NPs can not only enhance the chemosensitization of OSCC but also improve the radiosensitization of OSCC. Teraoka et al. have shown that the addition of gold NPs can enhance the effects of X-ray irradiation against oral cancer cells *in vitro*. The underlying cause of this cytotoxicity was the induction of apoptosis [78]. Gold NPs are much more efficient photon-thermal-energy converters and can be used for photothermal therapy (PTT). PPT is mediated efficiently by gold NPs that can powerfully absorb NIR light and efficiently convert into heat energy due to SPR. It is noteworthy that tumor cells are more sensitive to hyperthermia than normal cells, especially at temperatures above 42°C [79]. Liu et al. investigated a (podoplanin antibody) gold NPs-DOX system as a nanoplatform combining chemophotothermal therapy to obtain enhanced antitumor efficacy. Podoplanin-antibody-conjugated gold NPs can facilitate the accumulation of the drug and NPs in the tumor site through active targeting. The DOX release rate increased under the acid condition of endolysosomal compartments of tumor cells, which might be due to the disruption of the acid-sensitive amide bond between the PEGylated AuNPs and DOX [80]. In addition to EGFR-specific targeting, Melancon et al. have explored a multifunctional gold nanoshell coated with superparamagnetic iron oxide. This system can thermally induce tumor destruction and reduce thermal damage to surrounding normal tissues under an MRI-visible approach [81]. Nanoparticle-induced cytotoxicity was associated with autophagy-mediated mechanisms [82]. The use of upconversion NPs conjugated with Au nanorods can enhance plasmon-PDT [83, 84].

## 5. Magnetic Nanoparticles for Oral Cancer Diagnosis and Therapy

MNPs with various shapes and modifications (Figure 5(a)) exhibit high magnetic properties, good stability, biocompatibility, and biodegradability. There is a wide range of applications in magnetic resonance imaging (MRI), drug delivery systems, and hyperthermic treatment of various cancers including oral cancer (Figure 5(b)). To date, numerous different methods have been developed to synthesize MNPs, including coprecipitation, thermal decomposition, microemulsion, hydrothermal, sol-gel, combustion, and polyol syntheses. [85, 86]. However, due to the potential of uptake by the RES and agglomerated tendency, the applications of MNPs remains limited. Polymeric coatings provide a barrier to avoid uptake by the RES and prevent nanoparticle agglomeration [23].

### 5.1. Magnetic Nanoparticles for Oral Cancer Diagnosis

Magnetic resonance imaging (MRI) is one of the most useful noninvasive imaging modalities utilized in clinical medicine today. MNPs are being actively investigated as MRI contrast agents and can help to refine proton relaxation, gradually, developing as useful probes as a contrast for both in the applications of medical and biological diagnostics [87]. MNPs also can be selectively injected into the tumor site without penetrating other organs [88]. The next generation of active targeting MNPs has the potential to provide significantly improved tumor detection and localization by utilizing the unique molecular signatures of these diseases.

### 5.2. Magnetic Nanoparticles for Oral Cancer Therapy

MNPs, as one of the most promising targeted drug delivery systems, have been applied to accumulate drugs specifically to the tumor site under the control of an external magnetic field (Figure 5(c)). However, the nonporous surface of MNPs is an issue in the application of the drug carrier. To overcome this shortcoming, Zhang et al. have proposed an MNP system synthesized by the solvothermal method, and the surface of MNP was modified by polyacrylic acid (PAA) to increase bleomycin (BLM) loading amounts. BLM-MNPs were constantly gathered into tumor tissue under the magnetic field and inhibited their growth by releasing BLM locally and steadily [89]. Recently, the recent study in NP-based gene therapy has given hope for cancer treatment because RNA interference (RNAi) takes part in the gene silencing process in eukaryotes and can be triggered by small interfering RNA (siRNA) and microRNA (miRNA). Therefore, MNPs could be designed to target these genes. Inhibition of both B-cell lymphoma-2 (BCL2) and Baculoviral IAP repeat-containing 5 (BIRC5) leads to apoptosis. Jin et al. have designed an siRNA-targeting BCL2 and BIRC5 delivery system based on the Fe_3_O_4_ NPs. MNP coating with the polyethyleneimine (PEI) provided a positive charge, which is necessary for siRNA capture and plays the role of gene silencing after the cellular uptake [90]. Targeting to the human-TRAIL gene, Miao et al. have used PEI-modified Fe_3_O_4_ NPs driven by the hTERT tumor-specific promoter to induce apoptosis [91]. Cancer cells show more sensitivity to hyperthermia compared with normal cells. PTT can inhibit the proliferation process of tumor cells and induce degeneration and necrosis of the tumor cells. Although gold-nanoparticle-mediated PTT can kill oral cancer cells, PPT is generally suitable for the therapy of superficial tumors. Magnetic fluid hyperthermia can generate heat under an alternating magnetic field (AMF) through magnetic vector rotation and physical rotation, inducing irreversible cellular damage and apoptosis of cells. Su et al. have explored superparamagnetic iron oxide NPs conjugated with anti-CD44 antibody to target CD44, a well-characterized oral carcinoma biomarker leading to the immune escape of cancer cells [92]. Legge et al. have produced biocompatible silica-coated magnetic iron oxide NPs conjugated with antibodies to target integrin *α*v*β*6, an overexpressing oral squamous cell carcinoma biomarker associated with poor prognosis [93]. Both research results have shown that the growth of tumors has been inhibited by targeting magnetic hyperthermia without damaging surrounding normal tissues. Furthermore, thermochemotherapy plays a new and important role in anticancer treatment. Sato et al. have utilized ferucarbotran (commercial-grade superparamagnetic iron oxide) combined with cisplatin to state that combinations of magnetic hyperthermia with chemotherapy may be more effective than either hyperthermia or chemotherapy alone; moreover, thermochemotherapy can reduce the effective dosage of cisplatin [94].

## 6. Quantum Dots for Oral Cancer Diagnosis and Therapy

Quantum dots (QDs) are semiconductor nanocrystals composed of elements belonging to group II-IV, group IV-VI, or group III-V, which usually range from 1 to 10 nm in diameter [33]. QDs possess a high intensity of fluorescence, narrow emission spectrum, wide absorption spectrum, and wide excitation spectrum from ultraviolet to NIR (or between 450 and 850 nm) (Figure 6(a)). QDs can not only be applied as probes or carriers for drug delivery in cancer therapy but also can generate reactive oxygen intermediates/species (ROIs/ROS) or produce heat under irradiation to kill cancer cells [95].

### 6.1. Quantum Dots for Oral Cancer Diagnosis

QDs have more excellent optical features than traditional organic fluorescence materials due to their unique quantum size and surface effects. Zhao et al. have labeled Tca8113 cells by using QDs (goat anti-rabbit Qd_655nm_-igG) and the FITC labeling technique, observing that QDs have more outstanding fluorescence intensity and photostability than FITC and are more suitable for long-term dynamic observation of cell physiological changes [97]. Recently, the excellent optical properties of QDs have been widely developed for the diagnosis of cancer cells. For instance, Yang and Chen have fabricated EGFR-antibody-conjugated QD800 (QDs with a maximal emission wavelength of 800 nm) for the targeting and in *vivo* imaging of human buccal squamous cell carcinoma cell line (BcaCD885) in an OSCC animal model, and QD800 has strong penetration in tissues, which is suitable for visible fluorescence imaging [98].

QDs have been used to develop multifunctional nanoparticle probes by conjugating them with molecular biomarkers. These QDs probes can be employed to detect the expression of molecular biomarkers in oral cancer cells. For instance, Xue et al. have studied the formation of Caveolin-1 (Cav-1) in carcinogenesis and the development of tongue squamous cell carcinoma by semiconductor QDs immunofluorescence histochemistry (QDs-IHC). The result has suggested that Cav-1 protein is an oncogene in the carcinogenesis and development of tongue squamous cell carcinoma [99]. Besides, it is a major challenge when cells are at such extremely low amounts of nucleic acids and protein, which requires QDs with high binding specificity of target molecules for high-sensitivity detection. Xue et al. have used QDs in situ hybridization (QDISH) to examine the connection of OSCC and human papillomavirus (HPV), and the result has indicated the sensitivity was higher by QDISH than that by ISH [100].

In addition, biosensor based on QDs is a significant development that could aid certain biomarker detection in recent years. Xu et al. have developed a new electrochemical method to detect interleukin-8 (IL-8) by adding DNA-templated CdTe/CdS QDs (DNA-QDs), and target IL-8 are treated with tris (2-carboxyethyl) phosphine (TCEP) to obtain active thiols (SH) and then recognized and separated by magnetic beads (MBs). Thereafter, anti-IL-8@MBs are easily coupled with DNA-QD *via* the Michael addition reaction between the active thiol and the maleimide group. Therefore, it is a simple and effective way to test IL-8 by tracking the electrochemical responses of DNA-QDs [101].

### 6.2. Quantum Dots for Oral Cancer Therapy

The present study sought to develop a QD-based (goat anti-mouse QD_525nm_-IgG and goat anti-mouse QD_655nm_-IgG) method for long-term dynamic observation of the physiological changes of heat shock protein 70 (HSP70) and heat shock factor 1 (HSF-1) in SCC-25 cells induced by heat shock and to explore strategies to influence the impact of activation of HSF-1 and the accumulation of HSP70 in oral cancer [102].

Carbon QDs (CQDs) are newly developed fluorescent NPs and are made from carbon, ensuring extraordinary biocompatibility and stable fluorescence. Das et al. have synthesized an N-doped mesoporous hollow CQD (NCQD) with good thermal conversion efficiency and excellent fluorescence imaging property that can be used to trace the curative response of PTT [103]. Graphene quantum dots (GQDs) are another type of CQDs. Wei et al. have prepared a polyethylene-glycol-GQDs-Pt (GPt) nanocomposite for specific delivery of Pt to OSCC cells (Figure 6(b)). They demonstrated that GPt could greatly improve the chemotherapeutic efficacy for OSCC in both normoxia and hypoxia conditions [96].

## 7. Polymeric Nanoparticles for Oral Cancer Diagnosis and Therapy

Polymeric NPs are prepared by using natural polymers and synthetic polymers and encapsulate drugs for cancer therapy. They can be classified into two main types: nanocapsules and nanospheres (Figure 7) [104]. Active pharmaceutical ingredients can be encapsulated within the vesicular cavity or enclosed by the solidified polymeric shell in the nanocapsulate and be trapped within the sphere center or adsorbed at the mass surface in the nanosphere, respectively. Polymeric NPs are widely applied owing to their favorable features in terms of simple elaboration and design, good biocompatibility, a broad structure variety, and noticeable bioimitative characteristics [105–107].

### 7.1. Polymeric Nanoparticles for Oral Cancer Diagnosis

Polymeric NPs can be used as the contrast agent for the targeted photoacoustic imaging [108]. Yang et al. have reported a high-performance nanoparticle for fluorescent endoscopic detection of oral cancer. Folic-acid-conjugated chitosan NPs can enhance nanoparticle endocytosis by targeting folate receptors on oral cancer cells. The N-succinyl chitosan (SCHI) polymer with negative charge can enhance the 5-aminolevulinic acid (5-ALA) releasing in oral cancer cells by decreasing the intensity between chitosan and the drug [109].

### 7.2. Polymeric Nanoparticles for Oral Cancer Therapy

Polymeric NPs have been developed as effective drug-delivery vehicles with the potential to overcome poor cell permeability. Chitosan NPs acted as promising cancer drug vehicles that can encapsulate ellagic acid [110], glycyrrhetic acid [111], cisplatin [112], curcumin [113], etc. for topical and local application to oral tumors, protecting anticancer drugs from biological deactivation. Additionally, using cationic chitosan as the polymeric NPs allows for electrostatic interactions between it and anionic mucin proteins. The mucoadhesive properties of chitosan can prolong residence time at the delivery site, favoring anticancer drug bioavailability. Other polymer NPs can also be used for drug delivery. Poly(lactic-co-glycolic acid) (PLGA) NPs loaded with docetaxel and administered locally to the tumor site show an increased antiproliferative efficiency [114]. Cisplatin-bounded N-vinylpyrrolidone/acrylic acid NPs were continually released into the head and neck cancer cells and had an anticancer effect [115]. Eudragit® E is a cationic copolymer that has been used to improve the poor solubility of silibinin [116]. Electrostatic interactions can mediate the form of multilayer NPs to deliver Sraf (an inhibitor of tyrosine kinases), exhibiting superior anticancer activities than free Sraf in the oral cancer cells [117]. Ligand-decorated NPs can specifically bind to and be efficiently internalized in receptor-overexpressed OSCC cancer cells [118, 119]. Besides, polyelectrolyte-assembling multilayer NPs (MLNPs) have been developed as a drug delivery system encapsulated with multiple drugs, such as cisplatin and chrysin. The combinational drug had a superior therapeutic effect compared to single-cisplatin-loaded MLNPs [120]. Furthermore, Li et al. have successfully developed a new polymer with a ROS-cleaving thioketal linker for targeted drug delivery [121]. Similarly, Wang et al. have designed a potent ROS-sensitive delivery system for chemophotodynamic therapy. DOX was conjugated to self-destructive polymeric micelles to execute drug release through a light-triggered ROS [122]. The embedment of cupreous complexes into chitosan NPs can greatly suppress the release of inner toxicity, which allows the PDT *in vitro* and *in vivo* [123]. However, activation of the epithelial to mesenchymal transition (EMT) in PDT can lead to tumor recurrence. Polyethylene-glycol-polyethyl-eneimine-chlorin e6 NPs have been designed to efficiently transfer Wnt-1 siRNA into the cytoplasm of OSCC cells under the action of PDT, inhibiting the Wnt/*β*-catenin signaling pathway that is crucial to the EMT [124]. PEG-PCL-C3-indocyanine green (ICG) NPs were successfully prepared to serve as anticancer agents in combined PTT and PDT under laser irradiation, showing better therapeutic effects than PTT or PDT alone [125]. Recently, hyperbranched polymers are a new type of drug carrier, which can be used to prepare NPs with uniform size distribution. Li et al. have investigated the action of hyperbranched polymer- releasing drugs in acidic intracellular environments, TH287 (the MTH1 protein inhibiter) and anticancer drug sodium arsenite (an anticancer drug) can be loaded into hyperbranched poly(amine-ester) (HPAE) through electrostatic attraction and hydrophobic interaction, and TH287 renders more sensitive to drugs after inhibiting MTH1 in the tumor cell [126]. Hyperbranched polymers can also conjugate with photosensitizers such as chlorin(e6) and can be used in PDT on human tongue carcinoma CAL-27 cells [127].

## 8. Other Nanoparticles

Upconversion NPs (UCNs) can be used to improve the penetration depth limitations of conventional PDT. Lucky et al. have developed anti-EGFR-PEG-TiO_2_-UCNs for the targeted treatment of oral cancer cells. This system can be excited by deep-tissue-penetrating NIR light to induce cancer cell destruction in deeper tissues [128].

Carbon nanotubes can be developed as immunosensors for an oral cancer screening test. 3D high-aspect-ratio vertically aligned carbon nanotube arrays are arranged in a 2D interdigitated electrode (IDE) footprint by using chemical vapor deposition. The sensor demonstrated the ability to detect cancerous inhibitor PP2A (CIP2A) in saliva supernatant without the requirement for sample preconcentration or prelabeling techniques, showing higher biosensor sensitivity than the ELISA test kit. Moreover, this biosensor can save the total sensing time [129].

Wang et al. have fabricated a cationic polymer polyethylenimine-modified silica nanoparticle that could carry both MDR1-siRNA and DOX, which can efficiently transfect into human OSCC DOX-resistant cell line (KBV cells) in *vitro*. This system can block multiple drug resistance protein 1 (MDR1) expression to decrease multidrug resistance [130].

Metal-organic frameworks (MOFs) were employed as cisplatin and taxol drug delivery vehicles to enhance the sustained release and decrease the burst effect [131].

## 9. Conclusions

In this review, we summarized the recent advances of NPs for oral cancer diagnosis and therapy. The unique physicochemical features of NPs, including ultrasmall size, high reactivity, and tunable functional modification have been demonstrated to be accurate timely tools for oral cancer diagnosis and highly effective strategies for oral cancer treatment. The NPs provide a platform to enable visualization of oral cancer, selectively deliver therapeutic agents to tumors, and destruct tumors by different therapeutic techniques. Importantly, increasing attention will be paid to the hybrid systems, enabling NPs a flexible platform to achieve (bio)multifunctionality. Thereby, applying nanomedicine for the modern diagnosis and therapy of oral cancer is extensively anticipated.

Although the potential applications of NPs for diseases are currently very broad, the nanomedicine field is quite limited in applying nanoparticle technologies to the prevention and treatment of oral cancer. The research we described demonstrated excellent therapeutic activities in this review, mainly conducted *in vitro* or in preclinical models of oral cancer. Given the complex pathophysiology of oral cancer, such as abnormal hemodynamics, the pharmacokinetics and the biodistribution of therapeutic agents may vary, thereby yielding misleading findings. Thus, results from preclinical studies of new therapeutic agents for oral cancer must be viewed with a degree of skepticism. Moreover, the tiny size of NPs makes it easier for them to pass through cell membranes and other biological barriers. Therefore, NPs can be easily taken up into living organisms and cause cellular dysfunction. The improvement of the safety of these NPs cannot be ignored.

In addition, there is an urgent need to translate these preclinical outcomes into clinical applications. Successful completion of these clinical trials will set the foundation for further implementation of nanoparticle-based therapeutic and diagnostic products. Thus, there is considerable scope for the diagnosis and treatment of oral cancer based on NPs over the next couple of years.

## Figures and Tables

**Figure 1:** Nanoparticles for oral cancer diagnosis and therapy.

**Figure 2:** (a) The structure of liposomes. (b) The methods of liposome entering cancer tissue. (c) Diagnosis and therapy of liposomes.

**Figure 3:** (a) Multifunctional dendritic carrier with dual functions of diagnosis and treatment. (b) Nano-sar effectively suppressed invasion and metastasis of head and neck squamous cell carcinoma without systematic toxicities, Copyright 2018, Springer Nature [57].

**Figure 4:** (a) The geometries of gold NPs. (b) Diagnosis and therapy of gold NPs.

**Figure 5:** (a) MNP structures and coating schemes [23]. (b) MNP possessing various ligands to enable multifunctionality [23]. (c) The therapeutic effect of magnetic NPs under the control of an external magnetic field.

**Figure 6:** (a) The fluorescence emission properties of QDs can be modulated by changing their size. (b) Schematic illustration of a multifunctional anticancer platform against hypoxia-induced chemoresistance of OSCC [96].

**Figure 7:** The types of polymeric NPs. (a) The drug could be dispersed or covalently bound to the polymer matrix in nanospheres. (b) The drug could be encapsulated in the interior of the vesicular cavity or enclosed by the solidified polymeric shell in nanocapsules.

## Data Availability

The data supporting this review are from previously reported studies and datasets, which have been cited.
